# Prediction and Analysis of Corporate Financial Risk Assessment Using Logistic Regression Algorithm in Multiple Uncertainty Environment

This article has been retracted.

**DOI:** 10.1155/2022/2733923

**Published:** 2022-09-14

**Authors:** Xinyue Li, Saisai Yan, Jiajia Lu, Yanqiu Ding

**Affiliations:** College of Finance and Economics/Finance Teaching and Research Section, Shanghai Lida University, Shanghai 201600, China

## Abstract

Currently, the level of economic globalisation is expanding, which gives organizations more room to grow while also subjecting them to an increasing amount of pressure from the market. Companies are forced to deal with an increasing number of unclear aspects due to the unstable internal and external environments, which also increases the risks they confront. A management system for corporate financial risk is according to studies on early warning systems for financial risks. Its goals are to raise the standard of corporate financial management and boost economic advantages, identify concerns and potential hazards in the corporate financial management process, stop corporate financial crises in their tracks, and lessen the losses brought on by such crises. The financial risk management of the organization is predicted and examined in this research using the logistic regression model. The use of a logistic regression model allows for the simultaneous analysis of various risk factors, such as discrete and continuous variables, as well as the analysis of external variables' interactions and confounding. This method is suited for widespread usage in practice because it has shown exceptional outcomes in study that are 16.24% better than those of the conventional method.

## 1. Introduction

Under the environment of economic improvement and market opening, listed companies are developing rapidly and have broad prospects, but they are also under heavy pressure and fierce competition [1]. Enterprises are the most basic element of social production and the main force to promote economic improvement. Whether their improvement is healthy or not is not only related to their own destiny but also related to the national economy and national peace and security. The assumption of sustainable operation in classical finance theory is being relaxed in the face of the pressure from growing market competitiveness in the information economy, and the uncertainty faced by businesses is growing [2]. Due to financial crises, it is not uncommon for businesses to experience problems or even file for bankruptcy. Therefore, at any point in its business process, every organization must take into account early warning of financial crisis and collapse. It should begin to act as soon as anomalous indicators are discovered in order to prevent or lessen the harm to the business [3].

The low level of company financial management forms a sharp contrast with the high requirements of companies for financial management. It is an urgent task to establish a scientific financial management mode and improve the level of financial management [4]. At the same time, the operating status of the company will ultimately be reflected by financial indicators. Therefore, improving the financial management level can directly improve the overall management level of companies. It can be predicted that in the near future, most companies will gradually enter the stage of financial oriented corporate governance. In this economic environment, company financial management will become the core issue of corporate governance. The company operates as a whole, not only its scale, profit, and cost but also its overall consideration [5]. For example, in terms of capital operation, efficient operation can ensure the healthy improvement of companies and normal operation and investment; however, if the fund is not operated smoothly, it will lead to some situations such as insufficient debt repayment and disconnection of the capital chain, which will affect the normal production and operation of the company and aggravate the risk. The early warning of the financial crisis of the company has attracted much attention. In practice, in addition to the risk control of the credit of the lenders, the credit rating agencies must pay attention to the early warning of the financial crisis of the evaluated companies [6]. Financial risk early warning is based on the collection of financial conditions of listed companies, selecting representative financial indicator data, observing the impact of various financial indicators on the financial risk evaluation of listed companies, establishing models, predicting whether financial risks will occur in the future, issuing early warning signals to risk research objects in advance, helping companies find out the factors leading to risks as soon as possible, and taking corrective measures in the first time, to prevent greater losses [7]. Since post control is where the majority of conventional management theories and techniques go, managing risks quickly and effectively presents previously unheard-of obstacles. The financial risk early warning management theory, which is a novel idea that can track and foresee risks, is increasingly gaining favour with academics and businesspeople [8]. Financial risk develops through a complex process. It has internal relationships with all of the company's functional departments and is tightly tied to each step in the company's operational chain. Furthermore, the development of financial risk is a lengthy process that progresses from a quantitative to a qualitative alteration. The sooner it is identified and dealt with, the better for the business's secure financial operations [9]. Companies must continuously develop the financial security system and timely monitor their financial risks if they want to maintain the sustainability of economic growth and establish the market competitive advantages of financing and investment. The company must also establish and improve the financial crisis early warning indicator system from the perspective of high sensitivity and foreboding by closely relying on the inducement of financial crisis in order to prevent the occurrence of financial crisis, diagnose the crisis signal as early as possible, and take appropriate measures to eliminate the crisis in its embryonic stage [10]. We may also predict that there will be a substantial market for financial risk monitoring and crisis warning, which will support the development of in-depth study in this area.

A sound financial risk early warning system can detect the abnormal changes in the financial situation of companies as early as possible and analyze the causes, so as to effectively predict the signs of financial risks, enable company operators to take relevant preventive measures as soon as possible before the deterioration of financial risks, and eliminate the crisis in the bud [11]. Therefore, theoretically speaking, financial risk early warning is a powerful means for companies to prevent financial crisis and plays a very important role in the healthy improvement of companies. The innovation of this paper lies in (1) introduces the financial risk prediction. In this article, the logistic regression model is used to predict and analyze financial risk management. The complete text therefore focuses on predicting financial risk. We must now explain how to predict financial risk. (2) Introduces data mining (DM) and financial risk prediction. Next, we will explain the advantages of DM technique in financial risk, so that readers can have a general understanding of it. Otherwise, if the reader knows nothing about it, he will not know what we are talking about. (3) The method and results are introduced. Here, we introduce the methods and results of this paper. In this way, readers can participate in our research, so that they can have a better understanding of this study. Lead the reader into the research of this article.

## 2. Related Work

Zhu et al. suggested to select factor analysis and probability statistical analysis methods in the analysis of the company's business performance, select 15 financial indicators reflecting the company's profitability and solvency, analyze the average data, evaluate the overall business performance of the industry, analyze the reasons for this situation, and put forward corresponding countermeasures [12]. Phung et al. argued that the ratios of net profit to shareholders' equity and shareholders' equity to liabilities play a significant role in the early warning study's ability to anticipate company risk [13]. Sun and Lei proposed to develop a logistic regression and multiple discriminant analysis-based financial risk early-warning model using the company's financial data as variable indicators. According to empirical studies, the model is very capable of differentiating the company's financial status [14]. On the basis of earlier research, De proposed that the risk early warning model be upgraded and that 28 index data from two groups of companies be chosen. The findings demonstrate the effectiveness of the three measures for early warning and forecasting [15]: liabilities/total assets, cash flow/total liabilities, and total net income/total assets. According to Duprey and Klaus, the multivariate discriminant analysis prediction model can only categorise whether the sample company is experiencing a financial failing crisis and cannot calculate the likelihood of a crisis [16, 17]. Huang and Wang said that the model she created could ascertain the company's state and that operators were not required to have advanced professional skills in order to assess the company's health [18]. Zhu et al. suggested using univariate and regression analysis to construct a financial crisis early warning model using four different types of audit reservations and two financial ratios. According to the findings, only “reservations with questions about continued operation” and “reservations in other forms” in the multivariate model can reliably anticipate the financial crisis [11]. The other two types of reservations do not. For the SC Group's financial early warning model, Pompella and Dicanio recommended integrating the logistic regression method with the factor analysis method to increase the model's accuracy [19]. Qu and Li suggested that the addition of annual cumulative excess return of nonfinancial indicators and auditor's opinions improved the prediction accuracy of the model [20]. Zhu and Liu suggested that there are not only financial indicators but also nonfinancial indicators that affect the evaluation of the company's business performance. Taking nonfinancial indicators into account can more effectively evaluate the company's business performance. However, due to the nonoperability of nonfinancial indicators, it is still difficult to apply them [21]. Bao and Lin proposed to apply the multivariate linear research method to the financial risk early warning for the first time, adopt the statistical analysis method, and finally build the *Z* model with the result of minimum error judgment [22].

The development of a company's financial risk early-warning model is crucial to the functioning of the business and has a significant impact on the management strategy of managers and financial personnel. One of the most important and harmful hazards in business is financial risk. It will be challenging for businesses to escape the nightmare of bankruptcy if it is not promptly informed about and avoided. The development of financial early warning models is crucial for the running of businesses and has a significant influence on the management strategies used by managers and financial personnel. This study examines financial risk management prediction and analysis using a logistic regression model, which is very important.

## 3. Data Mining and Financial Risk Prediction

### 3.1. Financial Risk Forecast

The word “risk” comes from western economic theory. It refers to the change degree of various results that may occur in a certain period of time and under certain conditions. It is a potential possibility and an objective existence, which is also the reason why people cannot predict the occurrence of risk. Risk is a neutral term. There are many explanations for it in the academic circles. It generally refers to the degree of change of various results that may occur in a certain action under certain conditions and within a certain period of time. Its magnitude changes with time. It is caused by the uncertainty of the event itself, and it is objective. The dual nature of risk can bring excess profits or losses to companies. Broadly speaking, we think that the so-called financial risk refers to the loss caused by the difference between the financial income and the expected income in the company's operation under the influence of many uncertain factors. Therefore, companies attach importance to risk research and try to make a trade-off between risk and benefit. However, investors pay much more attention to unexpected losses than unexpected gains. Therefore, risk research focuses more on adverse aspects, and it is customary to equate risks with losses. There are also changes in the economic environment that will directly affect the financial affairs of listed companies. For example, the regional economic improvement is unstable, the overall social economic level changes, the industrial economic environment changes, and the tariff policy changes.

In the latter-day market economy, every company is faced with various risks from time to time in the process of establishment to growth, of which the most prominent are business risks and financial risks. Any problem in any link of the company's operation may cause this risk to turn into loss and reduce the profitability and solvency of the company. There is also a limited viewpoint that says a company's financial risk is the possibility that it will not have the money to pay its debts on time. According to this perspective, the financial risk is a result of the operation's debt and is brought on by the repayment of past-due loans or the repayment of past-due principal plus interest. Financial risk will not exist for the company if there is no debt, meaning that its operating capital is derived from investors' investments. The financial risk that businesses face extends beyond the extent of their financing activities, according to the perspective of financial early warning. Inappropriate distribution, operation, and investment activities may also expose businesses to danger. To increase the competitiveness of businesses and reduce financial risks, managers should develop numerous coping mechanisms for changing economic environments. Company financial operations include four parts from the entire process of a company's capital movement: finance activities, investment activities, operating activities, and income distribution activities. All of a company's financial activities fall under these four interconnected, constrained, and independent categories. Financial risk is a typical economic risk that has attracted a lot of interest in both theoretical and operational study.  Figure 1 displays the chart of the fund movement.

The management of financial risk is closely related to the improvement of companies, and many well-known companies suffer economic losses caused by financial risk due to poor management and even cannot escape bankruptcy. The premise of financial risk is commodity production and commodity circulation. There are many reasons for the financial risk of Chinese companies, including controllable and uncontrollable and internal and external. The specific reasons for the formation of different types of financial risk are different. Many of the external factors that cause the financial risk of the company are unpredictable, and the company can only respond passively. However, some internal controllable factors, such as improper operation and management, have a more direct impact on the financial risk of the company. Under the market economy environment, the financial risk of companies is inevitable. Any link of production and operation of a company is a market behavior. Financing needs to rely on the market, and production and sales should be adjusted according to market changes. There are many questions involved in the financial activities of companies, which are all over the whole process of company activities, for example, the proportion of self-owned funds to borrowings in company financing and the related liability management questions, the diversified investment questions in company investment, the proportion questions in company profit distribution, the inventory management and accounts receivable management in the daily asset management of companies, and so on.

### 3.2. Data Mining for Financial Risk Prediction

The rapid improvement of economy and the rapid improvement of science and technique jointly promote mankind to enter an era of information explosion. The improvement of companies is under the complex market environment system, which leads to many uncertainties in the improvement of companies. These uncertainties will lead to financial risks of companies.

The emergence of the Internet era also heralds the big data era, or the era of vast data. A significant amount of data has been produced in the business process due to the rising automation of corporate business operation processes. These data and the knowledge derived from them are the companies' priceless wealth since they accurately reflect the fundamental circumstances of business activity. However, a common problem faced by all companies is that the amount of company data is very large, and the really valuable information is very small. In the face of such a large amount of data, traditional data analysis methods, such as data retrieval and statistical analysis, can only obtain the surface information of the data, but cannot obtain its internal and deep-seated information. In addition, with the improvement of global economic integration, the financial environment of companies has changed dramatically, and the financial risks faced by companies are more diversified and complex. At the same time, the harm caused by financial risks to Chinese companies is also deepening. However, the traditional financial index analysis is based on historical data and basic regression analysis, which has certain limitations for the prediction of future uncertain factors. DM includes a series of technologies aimed at finding useful but undiscovered patterns from data sets. The purpose of DM is to model decision-making, that is, predict future behavior according to the analysis of past activities. This is also the most attractive place of DM, that is, it can establish prediction models instead of retrospective models.

Under the data background, it is easier and faster for people to obtain data, but they are still faced with the confusion of too much data and too little useful information. People are eager to find a tool to quickly process a large number of different types of data in a short time. In fact, it can be seen that what companies lack is not data, but tools for how to process and analyze data, so that massive data can play its due value, which requires the help of big DM technique. Big data helps people realize their desire to convert all the running things into data and store them. DM technique can filter and extract useful information from a huge amount of data, build an intelligent analysis system, and draw conclusions with decision-making reference value. Traditional financial analysis is mainly based on the historical data of financial statements. This analysis is an evaluation of past work and results, rather than a prediction of the future. In order to develop, companies should pay more attention to the future rather than the past. Therefore, traditional financial analysis is one-sided and cannot predict the future. The DM structure is shown in Figure 2.

Science, technology, and economy are constantly changing, and huge data are being collected and stored by companies. The traditional financial analysis method is more and more unsuitable for the present society, especially its one sidedness and lag cannot meet our needs. So we urgently need to apply data mining to financial analysis. With the progress of information technology, in daily life, enterprises will produce a large amount of financial data every day, and the requirements of leaders for financial decision-making information are also increasing. At this time, the traditional financial analysis method is definitely unable to meet their needs. Big data mining technology perfectly solves this problem. It can synchronously update the financial data into the system according to the preset model and process and then use the big data technology to realize analysis, which is fast and accurate, and at the same time, it can save huge labor costs.

## 4. Methods and Results

### 4.1. Logistic Regression Model

In recent years, companies have been involved in financial crisis and even bankruptcy from time to time. The number of bankruptcy of global companies is on the rise and has a wide range. However, this means of credit sales will make the company bear the application risk of the other party, often resulting in the failure to collect the accounts receivable on time and in full, and many companies fall into the dilemma of “waiting for death without credit sales, looking for death with credit sales.” This requires that companies must fully understand their customers and, before cooperation, make financial early-warning assessment on their finances, so as to formulate a reasonable financial system and lock in the financial risks of companies.

Assume that there are two possibilities for the value of *Y*, namely, 0 and 1, where 0 represents the financial risk of the company and 1 represents the financial status of the company. In this case, the linear model *Y*_*i*_ = *β*_0_ + *β*_1_*X*_1_ does not conform to its assumptions, but *Y*_*i*_ is a distribution of 0 and 1, so its mean value has special meaning in the model, such as

(1) $$\begin{array}{c} P=\left(Y_{i}=1\right)=\pi_{i},P=\left(Y_{i}=0\right)=1-\pi_{i}. \end{array}$$

From this, the value of *Y* can be obtained:

(2) $$\begin{array}{c} E\left(Y_{i}\right)=1\times \pi_{i}+0\times \left(1-\pi_{i}\right)=\pi_{i}. \end{array}$$

The *π*_*i*_ value in the above formula represents the probability value. It is best to use a multiple logistic regression model. If a linear model is used, a series of influencing factors will be generated. According to the principle, the following formula is obtained:

(3) $$\begin{array}{c} P_{i}=f\left(\beta_{0}+\beta_{1}X_{i1}+\beta_{2}X_{i2}+\cdots +\beta_{n}X_{\text{in}}\right). \end{array}$$

Wherein

(4) $$\begin{array}{c} f=\frac{ex}{1+ex}. \end{array}$$

*Y*_*i*_ can be expressed in another way:

(5) $$\begin{array}{c} P\left(Y_{i}\right)=\pi_{i}y_{i}\left(1-\pi_{i}\right)1-y_{i}. \end{array}$$

The logarithm obtained by using the maximum similar function method for the likelihood function is

(6) $$\begin{array}{c} LnL=\overset{n}{\underset{i=1}{\Sigma }}y_{i}\ln\pi_{i}+\left(1-y_{i}\right)\ln\left(1-\pi_{i}\right), \end{array}$$

(7) $$\begin{array}{c} \pi_{i}=\exp\left(\beta_{0}+\beta_{1}X_{i1}+\beta 2X_{i2}+\cdots +\beta_{n}X_{\text{in}}\right)\Lambda +\exp\left(\beta_{0}+\beta_{1}X_{i1}+\beta_{2}X_{i2}+\cdots +\beta_{n}X_{\text{in}}\right). \end{array}$$

Companies should constantly strive to innovate as this is essential to achieving positive change. Companies find it challenging to profit from the scale economy and achieve scale benefits due to restrictions imposed by scale, skill, and money. The company's improvement will be aided by the financial early warning if the company's operators, investors, and creditors are able to conduct appropriate early warning analyses of the company's financial situation and render wise decisions regarding business operations, investments, and creditor rights.

Let *X* = (*X*_1_, *X*_2_, ⋯*X*_*p*_) denote the evaluation index of company financial risk, and the linear regression algorithm is to find the best linear combination of evaluation indexes:

(8) $$\begin{array}{c} W_{0}+W_{1}X_{2}+W_{2}X_{2}+\cdots W_{ip}X_{p}=W^{*}•X^{*T}. \end{array}$$

This linear combination is used to express the probability of whether the company has financial risk, where *W*^∗^ = (*W*_0_, *W*_1_, *W*_2_, ⋯*W*_*p*_) is the coefficient of the evaluation index *X*^∗^ = (1, *X*_1_, *X*_2_, ⋯*X*_*p*_). If *P*_*i*_ is the probability that the *i*th company in the sample has financial risk, *W*^∗^ should be obtained to make the best estimate of the following formula:

(9) $$\begin{array}{c} P_{i}=W_{0}+X_{i1}W_{1}+X_{i2}W_{2}+\cdots +X_{ip}W_{p}. \end{array}$$

In equation (9), the value range on the right side of the equation is (−∞, +∞), but the probability value between [0, 1] is desired on the left side. Therefore, it is better to perform function transformation on the left side of the equation, and any value between (−∞, +∞) can be taken. After the transformation, the risk assessment value of the sample point and the value range of the evaluation index combination can be the same. The logit transformation of pairs can achieve this goal, which is defined as

(10) $$\begin{array}{c} \log\left(\frac{P_{i}}{1-P_{i}}\right)=W_{0}+W_{1}X_{1}+W_{2}X_{2}+\cdots W_{P}X_{p}=W•X^{T}. \end{array}$$

The formula is logistic regression model.

The prediction of financial risk management is examined in this work using the logistic regression model. Particularly in the disciplines of medicine, social research, processing biological data, and other areas, logistic regression analysis is frequently utilised as an efficient data processing technique. The choice of the regression model, cost function, and likelihood function in logistic regression analysis is frequently correlated with a particular probability distribution or probability model. The original data can be suitably altered during data processing, with the aim of as closely aligning the model with the real dose-response relationship as possible. In addition, the covariate distribution's skewness and kurtosis coefficients are not very high to guarantee the stability of convergence. Model construction requires a high level of expertise, particularly cumulative model construction. The right model must be chosen and reasonably built in accordance with the actual questions and the unique conditions of the data in the application, all while having a thorough understanding of the theoretical background, characteristics, and probability assumptions of the model. Regression analysis must also use the effective cost function or likelihood function to ensure a reasonable regression effect.

### 4.2. Results and Discussion

Generally, the so-called early warning system is a system that informs a person, an organization, or even a country in advance of the dangerous situation, and should pay attention to the genes that may cause a crisis and take preventive measures in advance. Different early warning indicators have different priorities and different prediction conclusions. Therefore, financial early warning indicators should be effectively classified according to the nature of the field to be monitored, and important indicators that can best reflect the characteristics of financial activities should be listed separately. Only by ensuring that the financial personnel can grasp the information in the first time can the overall timeliness of financial risk early warning be ensured, so that there can be enough time to evaluate the risk and select the best treatment method. Enterprise financial risk early warning system is a system engineering and one of the subsystems of management early warning system. The financial risk early warning system needs to establish the corresponding early warning organization system and early warning analysis methods to help realize the management functions of decision-making, organization, and control and to realize the self-balance and self-improvement in the business process of companies. It can be seen from Figures 3–5 that the simulation results of this method are relatively stable.

Financial early warning system is a system based on company informatization, with financial data as the main monitoring object, which can monitor the potential risks in the business management activities in real time. The financial early warning indicators designed by companies must be highly sensitive and can sensitively sense the initiation of abnormal factors in financial activities. Only in this way can the financial situation be reflected in a timely, accurate, and scientific manner, so that the abnormal changes can be controlled and the changes in financial activities can always be kept within a reasonable confidence interval. The financial risk early warning system shall conform to the system principle. That is to say, the financial early warning system is required to have the characteristics of integrity, which can not only ensure that the function and order of the financial management subsystem are in a reliable and controllable state but also affect the operation of the corporate governance system, that is, the decision-making of the corporate governance authority. The function of financial early warning system refers to the internal function of financial early warning system. It can be seen from Tables 1–3 and Figures 6–8 that the method in this paper has achieved remarkable results, which is 16.24% better than the traditional method, and is suitable for wide use in practice.

By strengthening management, the company's financial early warning system helps it to some extent to define its position in the market and prevent financial crises from happening. On the basis of accuracy, the established financial risk early warning indicators should also be as straightforward to calculate as possible, have strong operability, and be able to directly or indirectly calculate all pertinent indicators in accordance with the mastered financial accounting information. To ensure that staff members can follow descriptions in subsequent forecasting tasks, it is preferable to write explanations in straightforward language. The financial early warning system should have dynamic properties, which means that it must be able to forecast the company's improvement trend and assist the organization in developing smoothly toward the desired goal. The financial early warning system should also possess properties like openness, pay close attention to external information and the impact of the external environment on the organization's operation, and improve itself at any time. An organization's financial status deterioration happens over time. Financial early warning systems must connect the past to the present, view the company's business operations as a dynamic process, and identify future improvement trends based on historical analysis in order to effectively monitor an organization's operations. Therefore, a real-time and dynamic information system must be established as opposed to the conventional lagging accounting reflection for the financial early warning system. For weighing the benefits and drawbacks of a company's financial risk early warning system, the stability principle is a crucial requirement. In general, it is possible to calculate the relative change range of the majority of financial early warning indicators; but, because of their high volatility, financial predictions are more difficult to make and have a lower accuracy.

## 5. Conclusion

Financial hazards are a constant concern for businesses. An extreme example of financial risk is a financial crisis. However, neither the occurrence nor the cause of a financial crisis happens overnight. It emerges gradually and keeps building up over time. Financial crisis arises when a company's financial risk reaches a specific level of accumulation. Any corporation may face financial risks in its financial management activities given the intense market rivalry. The company will suffer financial losses or financial difficulties or possibly a financial crisis if it is unable to identify and effectively address the current and potential risks in a timely manner. This will start a domino effect that will result in unknown disasters for creditors, stockholders, and other stakeholders. The degree of financial risk for the organization can be quickly understood if it is assessed and handled quantitatively, allowing the company managers to make informed decisions. These needs can be satisfied by the financial early warning system. This method is suited for widespread usage in practice because it has shown exceptional outcomes in study that are 16.24% better than those of the conventional method.

## Figures and Tables

**Figure 1:** Fund movement chart.

**Figure 2:** Data mining structure.

**Figure 3:** Comparison chart of production cost of the company.

**Figure 4:** Membership function diagram.

**Figure 5:** Change of loss function.

**Figure 6:** Change of training error.

**Figure 7:** Correlation analysis between simulation output and target output.

**Figure 8:** Training results.

**Table 1:** Change of training error.

	0	2	4	6	8	10
Traditional method	0.06	0.19	0.12	0.17	0.23	0.04
Methods in this paper	0.03	0.14	0.06	0.04	0.04	0.25

**Table 2:** Correlation analysis between simulation output and target output.

	0	0.2	0.4	0.6	0.8	1
Traditional method	0.69	0.55	0.56	0.25	0.07	0.15
Methods in this paper	0.78	0.19	0.65	0.67	0.69	0.54

**Table 3:** Training results.

	0	20	40	60	80	100
Traditional method	0.72	0.95	0.21	0.04	0.69	0.46
Methods in this paper	0.90	0.46	0.28	0.67	0.31	0.38

## Data Availability

The data used to support the findings of this study are available from the corresponding author upon request.
